# Inhibition of microRNA-214 promotes epithelial–mesenchymal transition process and induces interstitial cystitis in postmenopausal women by upregulating Mfn2

This article has been retracted.

**DOI:** 10.1038/emm.2017.98

**Published:** 2017-07-21

**Authors:** Jian-Wei Lv, Wei Wen, Chen Jiang, Qi-Bo Fu, Yin-Jun Gu, Ting-Ting Lv, Zhen-Dong Li, Wei Xue

**Affiliations:** 1 Department of Urology, South Campus, Ren Ji Hospital, School of Medicine, Shanghai Jiaotong University, Shanghai, China; 2 Department of Urology, Shanghai General Hospital, School of Medicine, Shanghai Jiao Tong University, Shanghai, China; 3 Department of Urology, Ren Ji Hospital, School of Medicine, Shanghai Jiaotong University, Shanghai, China

## Abstract

Our study aims to investigate the roles that microRNA-214 (miR-214) plays in the epithelial mesenchymal transition (EMT) process and the development of interstitial cystitis (IC) in postmenopausal women by targeting Mitofusin 2 (Mfn2). IC bladder tissues and adjacent normal bladder tissues were collected from postmenopausal women. Immunohistochemistry (IHC) staining was conducted. The target relationship between miR-214 and Mfn2 was determined by a dual luciferase reporter gene assay. Adipose-derived mesenchymal stem cells (ADMSCs) were extracted from postmenopausal rats and assigned to the blank, mimics, miR-214 inhibitors, mimics negative control (NC), inhibitors NC, Mfn2 siRNA, miR-214 inhibitors and Mfn2 siRNA groups. Exosomes secreted by transfected ADMSCs were instilled into the bladders of postmenopausal rats. The expression of miR-214 and Mfn2 mRNA and EMT markers was assessed by qRT-PCR and western blotting. It was confirmed that Mfn2 was the target gene of miR-214 in IC. Compared with the normal bladder tissues, miR-214 decreased, but Mfn2 increased in IC bladder tissues. Compared with the blank group, the expression of miR-214 and the expression levels of N-cadherin, Fibronectin, Twist1, Snail and Vimentin mRNA and protein increased, whereas the expression levels of Mfn2, E-cadherin and ZO-1 mRNA and protein decreased in the miR-214 mimics and Mfn2 groups. The expression of MiR-214 and the expression levels of N-cadherin, Fibronectin, Twist1, Snail and Vimentin mRNA and protein decreased, whereas the expression levels of Mfn2, E-cadherin and ZO-1 mRNA and protein increased in the miR-214 inhibitors group. Our findings indicate that the inhibition of miR-214 promotes the EMT process and contributes to bladder wall fibrosis by up-regulating Mfn2, thus leading to the occurrence of IC in postmenopausal women.

## Introduction

As a recurrent and chronic inflammatory condition of the muscular and submucosal layers in the bladder, interstitial cystitis (IC) is defined as a syndrome with multiple etiologies and is characterized by pelvic bladder pain related to urinary urgency, frequency, burning and suprapubic pain with bladder pressure at a low-to-moderate degree.^1^ Because of the complication of its symptoms, IC is also referred to as irritable bladder syndrome, leaky bladder syndrome, and painful bladder syndrome, which are common in postmenopausal women.^1, 2, 3^ The occurrence of IC ranges from 1 in 100 000 to 5.1 in 1000 among the general population worldwide.^1^ Therefore, it is important to investigate the cellular and molecular mechanisms of IC for its management in postmenopausal women.

MicroRNAs (miRNAs) are 22-nucleotide conserved small noncoding RNAs that can negatively modulate gene expression via mRNA cleavage or translational repression through base pairing with complement sequences in the 3′ untranslated location (3′-UTRs) of target genes^4^ and are highly involved in different biological processes, including cell growth, metabolism and development.^5^ Recently, increasing evidence has demonstrated that miR-214 is involved in the development and progression of bladder cancer.^4, 6, 7, 8^ One study indicated that IC/bladder pain syndrome (BPS) may contribute to bladder cancer (BC) and an increased risk of BC.^9^ Therefore, we predicted that there may be an association between miR-214 and IC. Further analysis suggests that miR-214 is able to target Mitofusin 2 (Mfn2) and mediate the fibrosis process.^10^ Mfn2, which was originally discovered in vascular smooth muscle cells, also participates in cell proliferation and apoptosis. Mfn2 has been shown to have tumor-promoting functions in human cancer and may be an important therapeutic target for the treatment of urinary bladder carcinoma.^11^

A number of experiments have shown that mesenchymal stem cells (MSC) possess an inherent capacity to not only improve ischemia-related organ dysfunction^12, 13^ but also attenuate the inflammatory condition and reduce the adaptive and intrinsic immunity^14, 15^ by repressing immunogenicity.^16^ Recently, adipose tissue has been recognized as a convenient MSC source. Adipose-derived mesenchymal stem cells (ADMSCs), which are similar to MSCs from the bone marrow, have also been indicated to possess an immunosuppressive capability and differentiation potential.^17^ One study investigated the clinically therapeutic efficacy of ADMSCs in acute IC in rats when combined with melatonin treatment.^1^ However, the mechanism of ADMSC functioning in the pathogenesis of IC is under-investigated. Therefore, our study aims to explore the roles miR-214 plays in the ADMSC epithelial mesenchymal transition (EMT) process and the development of IC in postmenopausal women by targeting Mfn2.

## Materials and methods

### Study subjects

From May 2012 to October 2015, IC bladder tissues and adjacent normal bladder tissues were obtained from 24 postmenopausal women at Renji Hospital, School of Medicine, Shanghai Jiaotong University. The bladder tissues were obtained by bladder augmentation, after which the IC bladder tissues and adjacent normal bladder tissue cells were extracted. The adjacent normal tissues were treated as the control group. The diagnosis of IC conformed to the diagnostic criteria issued by the National Institute of Diabetes and Digestive and Kidney Diseases (NIDDK).^18^ All experimental procedures were approved by the Ethic Committee of Renji Hospital, School of Medicine, Shanghai Jiaotong University, and informed consent was obtained from all subjects.

### Hematoxylin-eosin, Masson and immunohistochemical staining

The tissues were fixed in formaldehyde and underwent conventional dehydration, xylene induced- transparency, wax dipping and paraffin embedding. The serial sections were approximately 3 μm and divided into three sections. The first section underwent HE staining. The slice was dewaxed at 50 °C for 1 h, stained with hematoxylin for 10–30 min, washed with tap water, differentiated using 1% acidic alcohol, dehydrated using gradient alcohol, stained with 0.5% eosin alcohol, decolored using 95% alcohol, made transparent using xylene, sealed with a neutral balsam, observed and photographed under an optical microscope. The second section underwent Masson staining. The slice was dewaxed at 50 °C for 1 h, chromized and washed; the nucleus was stained with Regaud’s hematoxylin for 5 min; and the section was washed again, stained with Ponceau S acid fuchsin for 5 min, bathed in 2% glacial acetic acid, differentiated using a 1% phosphomolybdic acid aqueous solution for 5 min, stained with a light green solution for 5 min, bathed in 0.2% glacial acetic acid, dehydrated using gradient alcohol, sealed with a neutral balsam, observed and photographed under an optical microscope. The muscular tissues were stained in red, the cell nucleus was stained in purple, and fibrous tissue was stained in green. The third section underwent IHC staining to detect the expression of the Mfn2 protein. The slice was dewaxed at 50 °C for 1 h, hydrated, subjected to antigen retrieval using a pH 6.0 sodium citrate buffer (0.01 M), incubated in 3% hydrogen peroxide for 10 min to inactivate the endogenous enzymes, sealed in bovine serum albumin (BSA) at room temperature for 30 min, incubated with an anti-human Mfn2 antibody (1: 200, Santa Cruz Biotechnology, Inc., Dallas, TX, USA) at 4 °C overnight, rewarmed at 37 °C for 1 h, incubated with a goat-anti-rabbit IgG at 37 °C for 30 min, incubated again with a Streptomyces antibiotic enzyme reagent at 37 °C for 30 min, developed using diaminobenzidine (DAB) at room temperature for 3–5 min, re-dyed for cell nucleus staining using hematoxylin, sealed with neutral resins, observed and photographed under an optical microscope. The results were assessed according to Fromowitz *et al.*^19^ by two experienced physicians.

### Establishment of the postmenopausal mouse model and extraction of ADMSCs

In total, 80 adult female SD rats, weighing 220–285 g, were purchased from the Ministry of Experimental Animals of China Medical University, Beijing, China. The rats had free access to food. The rat model was established using the ovariectomized method. Adipose tissue was collected from the rats by liposuction, and the ADMSCs were separated. The human IC bladder tissue, adjacent normal bladder tissue and adipose tissue from the postmenopausal rats were washed with D-Hanks buffer solution to remove hemocyte and necrotic cells. The samples were digested by 0.2% collagenase type II for 1 h and washed with D-Hanks buffer solution to remove collagenases. Cells were collected by centrifugation. Then, the cells were adjusted to 2 × 10^6^ per ml, seeded into a medium containing 95% DMEM/F-12 (Thermo Fisher Scientific Inc., Waltham, MA, USA), 5% fetal calf serum (FBS) (Thermo Scientific, Logan, UT, USA), 20 ng/ml epidermal growth factor, 100 U/ml penicillin and 100 U ml^−1^ streptomycin, and incubated in a CO_2_ incubator (Heraeus Holding, Nao, Germany) at 37 °C. After 24 h, the solution was replaced, and the cells without adherence were aspirated. Then, a half volume replacement was conducted every three days. Once the cell fusion rate reached 70–80%, 0.25% trypsin was added for conventional digestion. The cells were subcultured at 1: 3. On the 10th day, the expression levels of miR-214 and Mfn2 mRNA were detected by quantitative real-time PCR (qRT–PCR). All of the animal experiments in our study conformed to the local principle of animal management and usage and followed the Laboratory Animal Management and Use Guide by the National Institutes of Health (NIH).

### Identification of ADMSC differentiation and exosome extraction

The ADMSCs of sixth-generation rats were seeded into a T25 culture bottle at a density of 2 × 10^4^ per ml and cultured overnight. The cells were randomly assigned to two groups when the cell fusion rate reached 70–80%. The medium was replaced with an osteogenesis-inducing culture solution (H-DMEM medium containing 100 nmol l^−1^ hexadecadrol, 10% FBS, 10 mmol l^−1^ β-glycerophosphate and 0.2 mmol l^−1^ vitamin C) and adipogenesis-inducing solution (high glucose DMEM medium containing 1 × 10^−6^ mol l^−1^ hexadecadrol, 10% FBS, 100 μg ml^−1^ isobutylmethylxanthine (IBMX) and 50 μg ml^−1^ vitamin C). The cells were continuously cultured, and the solution was replaced every three days. Alizarin red staining (osteogenesis) and Oil Red O staining (adipogenesis) were adopted to assess the differential ability of ADMSCs. The alizarin red staining was conducted as follows: ADMSCs were washed with phosphate buffered saline (PBS) twice on the 12th day after osteoinductive differentiation, fixed in 95% ethyl alcohol for 10 min, washed with double distilled water (DDW), treated with 0.1% alizarin red-Tris-HCl at 37 °C for 30 min, washed with DDW, dried, sealed and observed under an inverted microscope. The jacinth mineralized nodule was positive in the extracellular matrix. The Oil Red O staining was performed as follows: ADMSCs were washed with PBS on the 12th day after adipogenesis-induced differentiation, fixed in neutral formalin for 10 min, washed with DDW, stained with 500 μl Oil Red O liquid for 5 min, sealed with glycerinum and observed under an inverted microscope. In the cytoplasm, a round bright red lipid droplet was positive. The medium was replaced by serum-free DMEM/F12 48 h after culture. The supernatant was collected by centrifugation and filtered with a 100 000 MW filter membrane. The supernatant was concentrated from 200 to 1–2 ml, after which transmission electron microscopy was applied to observe and photograph the extracted exosomes. An exosome is a 30–100 nm vesicle that is secreted by the polycystic body in living cells to the outside via membrane fusion and can transfer multiple molecules between cells.^20^ The expression of antigen protein was detected by western blotting.

### Dual luciferase reporter gene assay

The IC cells were seeded into a 96-well plate and subcultured. Once the cell density reached 70%, the cells were randomly assigned into the following 4 groups: the miR-214 mimics+Mfn2-3′-UTR-WT group (A group; transfected with 100 nmol l^−1^ miR-214 mimics and the Mfn2-3′-UTR-WT plasmid), the miR-214 inhibitors+Mfn2-3′-UTR-WT group (B group; transfected with 100 nmol l^−1^ miR-214 inhibitors and the Mfn2-3′-UTR-WT plasmid), the miR-214 mimics+100 Mfn2-3′-UTR-MUT group (C group; transfected with 100 nmol l^−1^ miR-214 mimics and 100 nmol l^−1^ Mfn2-3′-UTR-MUT plasmid), and the miR-214 inhibitors+Mfn2-3′-UTR-MUT group (D group; transfected with 100 nmol/l miR-214 inhibitors and the Mfn2-3′UTR-MUT plasmid). All the plasmids were purchased from Shanghai Gene Pharmaceutical Technology Corporation, Shanghai, China. The cells were incubated in a CO_2_ incubator at 37 °C for 6 h. Fresh nutrient medium was applied for another 48 h of incubation. Then, the cells were lysed, 100 μl phospholamban (PLB) solution was added, and the cells were slowly shaken for 15 min and preserved at −80 °C refrigerator. A dual luciferase reporter gene assay was performed in strict accordance with the dual luciferase reporter gene kit (Vigorous Biotechnology, Ltd., Beijing, China). A fluorescein detection reagent (100 μl) was added to a 1.5-ml Eppendorf (EP) tube. A luminometer was used for 10-s detection (TD20/20: Turner Designs, Sunnyvale, CA, USA) after a 2-s prediction. Then, 20 μl cell lysis buffer was added, the solution was fully mixed, and the samples were placed in an illuminometer for the firefly luciferase activity reading. 1 × Stop and Glo solution (100 μl) was added and fully mixed, after which the luminometer was applied for the renal luciferase activity reading. The expression of the reporter gene is shown as the ratio between the firefly luciferase activity and the renal luciferase activity (Y/H).

### Cell transfection and grouping

The 6-carboxyl fluorescein (FAM)-labeled miR-214 mimics, miR-214 inhibitors, mimic negative control (NC), inhibitor NC, Mfn2 siRNA and blank plasmid dry powder (Shanghai Gene Pharmaceutical Technology Corporation, Shanghai, China) underwent transient centrifugation and were dissolved in ddH_2_O containing diethylpyrocarbonate (DEPC). The samples were stirred well in the dark, concentrated into 20 μmol/l working solutions (final concentration of 100 nmol l^−1^), and preserved at −20 °C. The ADMSCs at the logarithmic phase were obtained and randomly assigned to the following 7 groups: the blank group (A group; transfected with 100 nmol l^−1^ empty plasmid), the miR-214 mimics group (B group; transfected with 100 nmol l^−1^ miR-214 mimics plasmid), the miR-214 inhibitors group (C group; transfected with 100 nmol l^−1^ miR-214 inhibitors plasmid), the mimics NC group (D group; transfected with 100 nmol l^−1^ mimics NC plasmid), the inhibitor NC group (E group; transfected with 100 nmol l^−1^ inhibitor NC plasmid), the Mfn2 siRNA group (F group; transfected with 100 nmol l^−1^ Mfn2 siRNA plasmid), and the miR-214 inhibitors+Mfn2 siRNA group (G group; transfected with 100 nmol l^−1^ miR-214 inhibitors plasmid and 100 nmol l^−1^ Mfn2 siRNA plasmid). The transfections were conducted in accordance with the Lipofectamine TM 2000 (Invitrogen, Co., Carlsbad, CA, USA) reagent specification, 6 h after which a fresh nutrient solution was applied for another 48 h of culture. The samples were observed under a fluorescence microscope (NIKON Corporation, Tokyo, Japan) and an inverted microscope (OLYMPUS Corporation, Tokyo, Japan), and the transfection efficiency was calculated. Cell transfection efficiency (%)=cell numbers under the fluorescence microscope/cell numbers under an ordinary light microscope × 100. The transfected cells were obtained and filtered by a 100 000 MW filter membrane. The obtained exosome was divided two sections. One section underwent qRT-PCR to detect the miR-214 and Mfn2 mRNA expression levels. The other section was used to culture the adjacent normal bladder tissue cells for 10 days. qRT–PCR and western blotting were applied to detect the relative protein expression levels in the epithelial and mesenchymal cells in each group.

### Animal grouping

In total, 96 female postmenopausal SD rats (145–180 g) were obtained and had free access to food and water. The rats were randomly assigned to the following 8 groups: the blank group (A group; transfected with an empty plasmid), the miR-214 mimics group (B group; transfected with the miR-214 mimics), the miR-214 inhibitors group (C group; transfected with the miR-214 inhibitors), the mimics NC group (D group; transfected with the mimics NC), the inhibitors NC group (E group; transfected with the inhibitors NC), the Mfn2 siRNA group (F group; transfected with the Mfn2 siRNA), the miR-214 mimics+Mfn2 siRNA group (G group; transfected with the miR-214 mimics and Mfn2 siRNA), and the normal saline (NS) group (H group; perfused with NS). Rats in the NS group were anesthetized with PE-50, and the rats in the other groups were anesthetized with an intraperitoneal injection of 5% amobarbital sodium. After the rats were lubricated with aseptic paraffin oil, a catheter was inserted through the urethral canal to the empty rat bladder. Exosomes (0.5 ml per group) were injected into the rats’ bladders in the blank, miR-214 mimics, miR-214 inhibitors, mimics NC, inhibitors NC, Mfn2 siRNA and miR-214 mimics+Mfn2 siRNA groups, while NS (0.5 ml) was injected and stored in the rats’ bladders for 30 min in the NS group. All rats were treated three times a week for 1 month. The rats were killed with CO_2_ within 48 h after the last treatment. The bladder tissues were obtained via bladder augmentation. One part was fixed in formaldehyde, underwent conventional dehydration, became transparent using xylene, and underwent wax dipping, paraffin-embedding, HE staining, Masson staining and IHC staining. The relative protein expression levels of epithelial and mesenchymal cells in the bladder tissues in each group were detected by RT–PCR and western blotting.

### Real-time reverse transcription–PCR

Total RNA for real-time reverse transcription–PCR (qRT–PCR) was extracted using the TRIzol method; the relative primers are shown in Table 1. The total RNA was reverse transcribed to cDNA using a PrimeScript RT kit (TaKaRa, Shiga, Japan). A total volume of 10 μl was used with reaction conditions at 37 °C for 15 min in triplicate and an inactivation reaction at 85 °C for 5 s. The qRT-PCR reaction was conducted using a SYBR Premix Ex Taq II kit (Takara Bio, Kyoto, Japan) with glyceraldehyde-phosphate dehydrogenase (GAPDH) as the internal control. A total volume of 50 μl consisted of SYBR Premix Ex Taq II 25 μl, PCR upstream primer 2 μl, PCR downstream primer 2 μl, ROX Reference Dye (50 ×) l μl, DNA template 4 μl, and dH_2_O 16 μl. The ABI Prism 7300 system was utilized for the qRT-PCR. The reaction conditions were as follows: pre-denaturation at 95 °C for 15 min, denaturation at 95 °C for 15 s, and annealing and extension at 60 °C for 60 s (40 cycles). Finally, the FAM490 fluorescence intensity was assessed. The relative expression levels of mRNA in each group were calculated via the 2^−ΔΔCt^ method with GAPDH as the internal control as follows: ΔCt=Ct _target gene_−Ct _reference gene_ and ΔΔCt=ΔCt _experimental group_−ΔCt _control group_.

### Western blotting

The protein expression levels were detected using the BCA method with GAPDH as the internal control. An equivalent amount of protein was obtained for the SDS–PAGE, in which different molecular weight proteins were separated, and the gel was transferred onto a nitrocellulose membrane. The membrane was blocked with 5% skim milk for 1.5 h and incubated overnight with the following primary antibodies: CD63 (1: 1000, ab59479), HSP70 (1: 1000, ab2787), HSP90 (1: 1000, ab13492), E-cadherin (1: 10 000, ab40772), N-cadherin (1: 1000, ab18203), Fibronectin (1: 1000, ab2413), Twist1 (1: 50, ab50887), Snail (1: 1000, ab53519), Vimentin (1: 500, ab8978), and ZO-1 (1: 500, ab61357) at 4 °C. All of the primary antibodies were purchased from Abcam Public Limited Company, Cambridge, UK. The membrane was washed with PBS and incubated with a horseradish peroxidase (HRP)-labeled goat-anti-rabbit secondary antibody for 2 h. After washing with PBST at least 3 times, the membrane was exposed to the enhanced chemiluminescence (ECL) reagent and photographed with a gel imaging system (Bio-Rad, Inc., Hercules, CA, USA). The gray value of the bands was analyzed with GAPDH as the internal control. The relative protein expression was calculated using 2^−ΔΔCt^.

### Statistical analysis

The data were analyzed using SPSS 21.0 (SPSS, Inc.; Chicago, IL, USA). For pairwise comparisons, *t*-tests were used, and a one-way analysis of variance was conducted for the multi-group comparison. *P*<0.05 was considered statistically significant.

## Results

### Pathological observations of the human adjacent normal bladder tissues and IC bladder tissues

A pathological observation of the adjacent normal and IC bladder tissues was performed. The HE staining results showed that in the adjacent normal bladder tissues, there was a thick mucus layer, no edema in the lamina propria, abundant muscle fibers, clear detrusor muscle and no inflammatory cell infiltration in the muscle bundles. In the IC bladder tissues, there was a thinner mucosal epithelium, edema in the lamina propria, muscle fiber atrophy, slender hair-like muscle bundles and chronic inflammatory cell infiltration in the muscle bundles. These results indicated that chronic inflammation played an important role in the development of IC. The Masson staining results showed well-arranged smooth muscles, abundant muscle fibers in the bladder wall, plump cells (red) and a small amount of fiber deposition between the detrusor muscle bundles (green) in the adjacent normal bladder tissues, while disordered smooth muscles, detrusor atrophy (red), a larger number of fiber deposition between the muscle bundles (green) and abundant inflammatory cell infiltration (purple) were observed in the IC bladder tissues (Figure 1). These results implied that fibrosis was a vital pathological manifestation in IC bladder tissues. The results of the IHC staining and qRT-PCR indicated that the expression levels of Mfn2 mRNA and protein were higher but that the relative expression of miR-214 was lower in the IC tissues than those in the adjacent normal bladder tissues (Figure 2).

### Differentiation ability of ADMSCs and identification of exosomes

The ADMSC collected from the rat adipocyte was a fibroblast-like cell. On the 12th day after the induction of osteogenesis and adipogenesis, the ADMSC was stained with alizarin red and Oil Red O. All results were positive, indicating that ADMSCs of rats had both adipogenic and osteogenic differentiation abilities. The exosome was collected from the supernatant of the ADMSC culture medium. Western blotting was applied to assess the expression of the antigen, and the results indicated that CD63, HSP70 and HSP90 were positive. The exosome presented as a 40–100 nm utricle bubble structure under a transmission electron microscopy (Figure 3).

### Expression levels of miR-214, Mfn2 mRNA and EMT markers in normal bladder tissues, normal bladder cells treated with exosomes and IC bladder tissues

In normal bladder cells treated with exosomes and IC bladder cells, the expression of miR-214 and of E-cadherin and ZO-1 mRNA and protein significantly decreased, whereas the expression of Mfn2 mRNA and of N-cadherin, Fibronectin, Snail, Twist1 and Vimentin mRNA and protein increased compared with the expression observed in the normal bladder cells (all *P*<0.05). No significant difference was found between the normal bladder cells treated with exosomes and the IC bladder cells (*P*>0.05; Figures 4 and 5). The results showed that that exosome could promote the EMT process and lead to bladder wall fibrosis, further inducing the occurrence of IC.

### Mfn2 is the target gene of miR-214

The TargetScan online software was applied to predict the possible gene targeted of miR-214. It was found that a fragment of miR-214 nucleotide was complementary with Mfn2 at the 5′-UTR, which was a highly conserved sequence compared with the miR-214 series among many species, indicating that Mfn2 could be the target gene of miR-214 (Figure 6). To verify this result, the IC bladder cells were transfected with different plasmids. Compared with the Mfn2-3′-UTR-WT+miR-214 mimics group, Y/H significantly increased in the Mfn2-3′-UTR-WT+miR-214 inhibitors, Mfn2-3′-UTR-MUT+miR-214 mimics and Mfn2-3′-UTR-MUT+miR-214 inhibitors groups (all *P*<0.05). No significant difference was found among the Mfn2-3′-UTR-WT+miR-214 inhibitors, Mfn2-3′-UTR-MUT+miR-214 mimics and Mfn2-3′-UTR-MUT+miR-214 inhibitors groups (all *P*>0.05; Figure 7). These results implied that Mfn2 was the target gene of miR-214 in IC.

### Expression levels of miR-214, Mfn2 mRNA and EMT markers in the seven groups

The exosome was collected after transfection. Compared with the blank group, miR-214 expression increased, but Mfn2 mRNA expression decreased in the miR-214 mimics and Mfn2 siRNA groups. MiR-214 expression decreased, whereas Mfn2 mRNA expression increased in the miR-214 inhibitors group. There was no significant difference among the mimics NC, inhibitors NC, miR-214 mimics+Mfn2 siRNA and blank groups (Figure 8). The adjacent normal bladder tissues were treated with an exosome after the transfection. After 10 days of culture, qRT-PCR and western blotting were applied to assess the expression levels of the EMT markers’ mRNA and protein in each group. Compared with the blank group, the expression levels of E-cadherin and ZO-1 mRNA and protein decreased, whereas those of N-cadherin, Fibronectin, Twist1, Snail and Vimentin mRNA and protein increased in the miR-214 mimics and Mfn2 siRNA groups. The expression levels of E-cadherin and ZO-1 mRNA and protein increased, whereas those of N-cadherin, Fibronectin, Twist1, Snail and Vimentin mRNA and protein were down-regulated in the miR-214 inhibitors group. No significant difference was found among the mimics NC, inhibitors NC, miR-214 mimics+Mfn2 siRNA and blank groups (Figure 9). These results indicated that the inhibition of miR-214 and the over-expression of Mfn2 could promote the EMT process and lead to bladder wall fibrosis, further inducing IC.

### Influence of the exosome on the expression levels of Mfn2 and EMT markers

The IHC staining results showed that compared with the blank group, Mfn2 expression significantly decreased in the miR-214 mimics and Mfn2 siRNA groups. An increase in Mfn2 expression was observed in the miR-214 inhibitors group. No significant difference was found among the mimics NC, inhibitors NC, miR-214 mimics+Mfn2 siRNA, NS and blank groups (Figure 10). The qRT–PCR and western blotting results indicated that compared with the blank group, the expression levels of E-cadherin and ZO-1 mRNA and protein were up-regulated, whereas those of N-cadherin, Fibronectin, Twist1, Snail and Vimentin mRNA and protein down-regulated in the miR-214 mimics and Mfn2 siRNA groups. The expression levels of E-cadherin and ZO-1 mRNA and protein decreased, whereas those of N-cadherin, Fibronectin, Twist1, Snail, and Vimentin mRNA and protein increased in the miR-214 inhibitors group. There was no significant difference among the mimics NC, inhibitors NC, miR-214 mimics+Mfn2 siRNA, NS and blank groups (Figure 11). These results further confirmed that inhibiting miR-214 could up-regulate Mfn2 expression, promote the EMT process and lead to fibrosis of the bladder wall, thereby inducing the occurrence of IC.

## Discussion

This study aims to investigate the interaction between miR-214 and Mfn2 in the IC of postmenopausal women. The findings of our study demonstrated that by targeting Mfn2, the suppression of miR-214 expression is able to promote the EMT process and contribute to bladder wall fibrosis, thus leading to IC in postmenopausal women.

Our initial findings reveal that the main syndrome of IC is a chronic inflammation and fibrosis in the bladder, and Mfn2 is up-regulated while miR-214 is inhibited in the IC bladder tissues. IC patients are reported to have elevated urinary nerve growth factor (NGF) levels and chronic inflammation localized to the urinary bladder.^21^ Furthermore, intrafascicular fibrosis can serve as a positive sign for the diagnosis of IC.^22^ To the best of our knowledge, Mfn2 is considered an important regulator controlling cell proliferation and tissue fibrosis.^23^ As indicated by Guo *et al.*,^24^ the over-expression of Mfn2 induces apoptosis in multiple cancer cell lines and cultured vascular smooth muscle cells (VSMCs) as shown by DNA laddering and cell death, which proved the inhibitory role of Mfn2 in cell proliferation in *in vitro* and *in vivo* studies using VSMCs. Recent studies have shown that Mfn2 over-expression can result in various disorders, such as lung cancers and hypertension.^11, 25^ Moreover, several studies have also demonstrated that the down-regulation of miR-214 can be used to determine the diagnosis, progression and recurrence of bladder cancer.^6, 7^ Wang and his colleagues showed that there is down-regulation of miR-214 in bladder lesion tissues, suggesting that miR-214 could exert a tumor-suppressive influence in bladder cancer through directly down-regulating oncogene PDRG1, which may act as a promising indicator for prognostic and therapeutic interventions in bladder cancer.^4^ In addition, a previous study reported that there may be an association between BC and a prior diagnosis of IC/BPS and explained that IC could cause tissue injury and activate the inflammatory cells and that this chronic inflammation could induce the development of cancer.^9, 26^ Therefore, we predicted that miR-214 may be involved in IC. In our study, the dual luciferase reporter suggested that Mfn2 is the target gene of miR-214, which is consistent with the results reflected in the study by Bucha *et al.*,^27^ who reported that miR-214 can regulate mitochondrial morphology and the cell cycle by targeting Mfn2. Additionally, in accordance with our finding, Sun *et al.*^28^ identified Mfn2 as a direct target gene of miR-214.

Subsequently, when normal bladder tissues are treated with an exosome, the expression levels of Mfn2 and the EMT-related proteins significantly changed with increases in the expression of Mfn2, N-cadherin, Fibronectin, Twist1, Snail and Vimentin m-RNA and reductions in the expression of miR-214, E-cadherin and ZO-1 m-RNA. Thus, we hypothesize that the exosome is able to promote EMT and contribute to bladder wall fibrosis, resulting in IC. The exosome is identified as a kind of micro-vesicle that is derived from a wide variety of cells and can act as a membrane fragment with a size of approximate 60–120 nm.^29, 30^ Furthermore, exosomes are composed of different subsets of miRNAs that are dependent on the cell type from which they are secreted.^31^ According to Zhu *et al.*,^32^ by triggering the extracellular signal-regulated kinase 1/2 (ERK1/2) pathway, ADMSC-exosomes increased the expression of vascular endothelial growth factor (VEGF) in tumor cells, thus leading to tumor growth *in vivo*. N-cadherin, Fibronectin, Twist1, Snail, E-cadherin, Vimentin and ZO-1 are related proteins in the EMT process,^33, 34^ and the conversion of epithelial cells into EMT has been to promote the growth of fibroblast-like cells.^35^ Moreover, our study implies that after transfection, miR-214 was down-regulated, Mfn2 was elevated, and there were elevated expression levels of N-cadherin, Fibronectin, Twist1, Snail and Vimentin and decreased expression levels of E-cadherin and ZO-1, thus further confirming the changes in expression levels of the EMT-related proteins, the reduced miR-214 expression and the increased Mfn2 expression. Those results indicate that the suppression of miR-214 is able to promote the EMT process and further lead to IC by up-regulating Mfn2. Interestingly, when the exosome of each transfected group is injected into the bladder of a postmenopausal rat, chronic inflammation and fibrosis are observed, which further explains that the inhibition of miR-214 can enhance the EMT process in the pathogenesis of IC by targeting Mfn2.

In conclusion, our experiment offers evidence for the mechanism of IC in postmenopausal women. Our data suggest that miR-214 is inhibited and Mfn2 is elevated in IC bladder tissues and that Mfn2 is the target gene of miR-214. In addition, the suppression of miR-214 is able to promote the EMT process and contribute to bladder wall fibrosis, thus leading to IC in postmenopausal women, which provides a novel insight into IC treatment.

## Figures and Tables

**Figure 1:** Pathological characteristics of the normal bladder tissues and IC bladder tissues observed by HE and Masson staining (200 ×). HE, hematoxylin-eosin; IC, interstitial cystitis.

**Figure 2:** The relative expression levels of miR-214 and Mfn2 mRNA and protein in normal bladder tissues and IC bladder tissues detected by qRT-PCR and IHC staining. *P<0.05 compared with the normal bladder tissues. IC, interstitial cystitis; IHC, immunohistochemical; qRT–PCR, quantitative real-time PCR.

**Figure 3:** Differentiation abilities of ADMSCs and the identification of exosomes. Note: (**a**) ADMSCs stained with alizarin red after the osteoinductive differentiation; (**b**) ADMSCs stained with Oil Red O after the adipogenic differentiation; (**c**) Exosome protein expression detected by western blotting; (**d**) Exosome structure under the transmission electron microscopy (50 000 ×); ADMSC, adipose-derived mesenchymal stem cells.

**Figure 4:** The expression of miR-214 and Mfn2 mRNA in normal bladder cells, bladder cells treated with exosomes and IC bladder cells. *P<0.05 compared with normal bladder cells. IC, interstitial cystitis; 1, normal bladder cells; 2, bladder cells treated with exosomes; 3, IC bladder cells.

**Figure 5:** The mRNA and protein expression levels of EMT markers in normal bladder cells, bladder cells treated with exosomes and IC bladder cells. *P<0.05 compared with the control group; EMT, epithelial mesenchymal transition; IC, interstitial cystitis; 1, normal bladder cells; 2, normal bladder cells treated with exosomes; 3, IC bladder cells.

**Figure 6:** The highly conserved binding sites of miR-214 and Mfn2.

**Figure 7:** Expression levels of luciferase in the IC bladder cells at 48 h after the transfection in the four groups. Note: (**a**) Mfn2-3′-UTR-WT+miR-214 mimics group; (**b**) Mfn2-3′-UTR-WT+miR-214 inhibitors group; (**c**) Mfn2-3′-UTR-MUT+miR-214 mimics group; (**d**) Mfn2-3′-UTR-MUT+miR-214 inhibitors group; *P<0.05 compared with the Mfn2-3′-UTR-WT+miR-214 mimics group, IC, interstitial cystitis; MUT, mutant type; WT, wild type.

**Figure 8:** The expression levels of miR-214 and Mfn2 mRNA in exosomes after the transfection in the seven groups. *P<0.05 compare with the blank group. NC, negative control.

**Figure 9:** The mRNA and protein expression levels of the EMT markers in the normal bladder cells treated with exosomes in the seven groups. Note: (**a**) group, transfected with an empty plasmid; (**b**) group, transfected with miR-214 mimics; (**c**) group, transfected with miR-214 inhibitors; (**d**) group, transfected with mimics NC; (**e**) group, transfected with inhibitors NC; (**f**) group, transfected with Mfn2 siRNA; (**g**) group, transfected with miR-214 mimics and Mfn2 siRNA; *P<0.05 compared with the blank group. EMT, epithelial mesenchymal transition; NC, negative control.

**Figure 10:** The expression level of Mfn2 protein in rats detected by immunohistochemical staining in the eight groups. Notes: (**a**) group, transfected with an empty plasmid; (**b**) group, transfected with miR-214 mimics; (**c**) group, transfected with miR-214 inhibitors; (**d**) group, transfected with mimics NC; (**e**) group, transfected with inhibitors NC; (**f**) group, transfected with Mfn2 siRNA; (**g**) group, transfected with miR-214 mimics and Mfn2 siRNA; (**h**) group, normal saline; *P<0.05 compared with the blank group. NC, negative control.

**Figure 11:** The mRNA and protein expression levels of the EMT markers in the rats in the eight groups. Notes: (**a**) group, transfected with a blank plasmid; (**b**) group, transfected with miR-214 mimics; (**c**) group, transfected with miR-214 inhibitors; (**d**) group, transfected with mimics NC; (**e**) group, transfected with inhibitors NC; (**f**) group, transfected with Mfn2 siRNA; (**g**) group, transfected with miR-214 mimics and Mfn2 siRNA; (**h**) group, normal saline; *P<0.05 compared with the blank group. EMT, epithelial mesenchymal transition; NC, negative control.

**Table 1:** Primer sequences for qRT–PCR

*Gene*	*Sequence*
*miR-214*	
upstream	5′-AGCATAATACAGCAGGCACAGAC-3′
downstream	5′-AAAGGTTGTTCTCCACTCTCTCAC-3′
	
*Mfn2*	
upstream	5′-ATGTCCCTGCTCTTCTCTCGATGC-3′
downstream	5′-TCTGCTGGGCTGCAGGTACTGGT-3′
	
*E-cadherin*	
upstream	5′-CCCACCACGTACAAGGGTC-3′
downstream	5′-ATGCCATCGTTGTTCACTGGA-3′
	
*N-cadherin*	
upstream	5′-TGAAGTCCCCAATGTCTCCA-3′
downstream	5′-GCATCATCATCCTGCTTATCC-3′
	
*Fibronectin*	
upstream	5′-CCCCATTCCAGGACACTTCTG-3′
downstream	5′-GCCCACGGTAACAACCTCTT-3′
	
*Twist1*	
upstream	5′-GAGGCGCCCCGCTCTTCTCCTCTG-3′
downstream	5′-CGTCTGAAGAACGGCGCGAA-3′
	
*Snail*	
upstream	5′-GAATTCATGCCGCGCTCTTTCCTCGTCAG-3′
downstream	5′-CTCGAGCCTCGAGGGTCAGCGGGGACATC-3′
	
*Vimentin*	
upstream	5′-AGAACTTTGCCGTTGAAGCTG-3′
downstream	5′-CCAGAGGGAGTGAATCCAGATTA-3′
	
*ZO-1*	
upstream	5′-CAACATACAGTGACGCTTCACA-3′
downstream	5′-GACGTTTCCCCACTCTGAAAA-3′
	
*GAPDH*	
upstream	5′-GGTCACCAGGGCTGCTTTTA-3′
downstream	5′-GAGGGATCTCGCTCCTGGA-3′

Abbreviation: qRT–PCR, quantitative real-time PCR.
